The article "New Criteria Could Improve the Success Rate of Non-operative Management of Acute Appendicitis in Children" was retracted in 2023. Reasons: errors in the data; errors in the methods; errors in the results or conclusions.

# New Criteria Could Improve the Success Rate of Non-operative Management of Acute Appendicitis in Children

**DOI:** 10.7759/cureus.25857

**Published:** 2022-06-11

**Authors:** Osman Uzunlu, Incinur Genisol

**Affiliations:** 1 Pediatric Surgery, School of Medicine, Pamukkale University, Denizli, TUR

**Keywords:** appendectomy, nonoperative treatment, children, conservative management, appendicitis

## Abstract

Background: Most studies addressing non-operative management for acute appendicitis have focused on adults, and there are limited data available for children. We aimed to evaluate the results of successful non-operative management in children with acute uncomplicated appendicitis with our “additional criteria” and find which factors could be affecting the success rate and which cases could be candidates for non-operative management.

Materials and methods: A total of 54 patients who were diagnosed with acute uncomplicated appendicitis and received non-operative management were re-evaluated retrospectively. Defining uncomplicated appendicitis was based on the duration of symptoms (<24 hours), clinical history, and radiologic findings. The radiologic evaluation was based on ultrasonography and computed tomography. The patients received an intravenous antibiotic combination (sulbactam/ampicillin, gentamicin, clindamycin) for five days at the hospital; the treatment was completed after 10 days with an oral antibiotic combination (amoxicillin/clavulanate, metronidazole). The cases have a follow-up period of up to two years.

Results: The mean patient age and follow-up time were 13.0 ± 4 years and 41.6 ± 13 months, respectively. The mean leukocyte count, C-reactive protein (CRP), and appendix diameter values were 15.48 ± 6.4 × 109/L, 11.79 ± 24.5 mg/dL, and 7.76 ± 1.4 mm on admission, and 6.86 ± 12.4 × 109/L, 4.17 ± 10.3 mg/dL, and 5.82 ± 1.6 mm on the second day, respectively. This decrease in WBC/CRP values and appendix diameter was statistically significant (p < 0.001). None of the patients had an early failure, complication, or adverse event. Recurrent appendicitis occurred in only five cases (9%) that were treated by laparoscopic appendectomy during the follow-up.

Conclusion: Non-operative management for acute uncomplicated appendicitis in children regarding long-term outcomes with our criteria was satisfactory and initial success rates were excellent.

## Introduction

Acute appendicitis is the most common abdominal surgical pathology in children [1]. The standard therapeutic approach is appendectomy. Surgical intervention has some complications that can result in morbidity and mortality [2]. The surgical approach has been questioned for uncomplicated appendicitis in recent years, and antibiotic therapy has been proposed as an alternative treatment [3]. Non-operative management for acute appendicitis has been developed in adult cases and has been safely adapted for children over time. However, there have been only limited reports describing non-operative management among the pediatric population [4-16]. These studies have specific criteria and different outcomes. This study aimed to evaluate non-operative management for uncomplicated cases and find which factors could be affecting success rate and outcomes.

## Materials and methods

This is a retrospective descriptive study. After obtaining permission from the University Ethical Committee, Pamukkale University (E-60116787-020-149479), the records of 208 cases diagnosed with acute appendicitis from April 2016 to February 2020 were reviewed. A total of 154 out of 208 patients were managed surgically (77 open appendectomies and 77 laparoscopic appendectomies), and the rest (54 patients) were treated non-operatively. Of the non-operatively treated appendicitis cases, only those who completed their two-year follow-up were included in the study. Patients with complicated appendicitis, fever at the time of admission, signs of fecalith on radiologic evaluation, and a follow-up period of less than two years were excluded from the study.

Diagnosis of acute appendicitis

The diagnosis of acute appendicitis was based on history, physical examination, laboratory results, and radiologic evaluation. Radiologic scans were routinely used in suspected acute appendicitis cases. Ultrasound (US) is preferred as the first-choice imaging method. However, in cases where the appendix is not visualized ultrasonographically, a CT scan is performed. The appendix diameter higher than 6 mm, uncompressible appendix, and echogenicity of tissue around the appendix were confirmed as acute appendicitis in the ultrasonographic exam.

Definitions

Our inclusion criteria for non-operative management were defined as symptom duration of less than 24 hours, localized tenderness, no signs of fecalith on radiologic evaluation, and no fever at the time of admission (Table 1).

**Table 1:** Inclusion criteria for non-operative management in our study

Patient evaluation	Inclusion criteria for non-operative management
Symptom duration	<24 hours
Clinical history	No fever and no additional disease
Physical examination	Localized tenderness
Radiologic evaluation (Ultrasonography and CT)	Without fecalith and perforation

The symptom duration of longer than 24 hours, generalized tenderness on physical exam, and radiologically suspected complicated appendicitis cases (abscess, phlegmon, irregular appendix wall) were managed operatively.

Treatment protocol

The non-operative management option was applied to those who did meet the criteria for non-operative management. Oral intake was not permitted during the first 24 hours of antibiotic treatment and hydration was provided by intravenous (IV) crystalloid solutions. The IV antibiotic protocol was ampicillin-sulbactam (150 mg/kg/day, divided into four doses), gentamicin (5 mg/kg/day, divided into two doses), and clindamycin (40 mg/kg/day, divided into four doses). All cases were evaluated by a physical examination at 12-hour intervals. For the patients who responded to antibiotic treatment after 24 hours, oral feeding was initiated. IV antibiotic duration was five days in all cases at the hospital, and all patients were discharged from the clinic with an oral antibiotic regimen (amoxicillin/clavulanic acid and metronidazole). Total antibiotic duration (IV and oral) lasted for 10 days.

Follow-up

All cases were re-evaluated by laboratory investigation and radiological examination. All blood samples and the US were repeated on the second day of the treatment. All of the patients were re-evaluated only by a physical exam on the second and seventh days of discharging at the outpatient clinic. Additional radiologic and laboratory screenings were not repeated at the outpatient clinic.

Ethical statements

All procedures performed in this study were in accordance with the ethical standards of the institutional and/or national research committee and with the 1964 Helsinki Declaration and its later amendments or comparable ethical standards. The parents were informed about the treatment protocol and complications. Informed consent was obtained from all individual participants included in this study.

Statistical analysis

Statistical analyses were performed using the Statistical Package for Social Sciences (SPSS) version 22.0 (IBM Corp., Armonk, NY). Statistics are presented as weighted mean ± standard deviation. The Kolmogorov-Smirnov test was performed to assess normal distribution. Parametric variables were analyzed by independent t-test and non-parametric variables by Mann-Whitney U test. The homogeneity of variance was determined by Levene's test. The level of statistical significance for descriptive statistics was set at p < 0.05.

## Results

The mean patient age was 13.0 ± 4 years (range: 4-17 years). A total of 29 (54%) cases were males and 25 (46%) were females; the male-to-female ratio was 1.16. The follow-up period of the cases ranged from 24 to 69 months, and the mean follow-up time was 41.6 ± 13 months.

Initial white blood cell (WBC) and C-reactive protein (CRP) levels at admission were 15.48 ± 6.4 × 10^9^/L and 11.79 ± 24.5 mg/dL, respectively. On the second day of treatment, the control results of WBC and CRP were 6.86 ± 12.4 × 10^9^/L and 4.17 ± 10.3 mg/dL, respectively (Table 2). This decrease in WBC and CRP values was statistically significant (p < 0.001).

**Table 2:** Laboratory and radiologic results

	At the time of admission	On the second day of admission	P-value
WBC (x10^9^/L)	15.48 ± 6.4	6.86 ± 12.4	0.001
C-reactive protein (mg/dL)	11.79 ± 24.5	4.17 ± 10.3	0.001
Appendix diameter (ultrasonography) (mm), n: 25/54	7.76 ± 1.4 (6-11)	5.82 ± 1.6	<0.001
Appendix diameter (computed tomography) (mm), n: 43/54	8.66 ± 2.0 (6-13)		

All cases were evaluated by the abdominal US at admission. US examination was repeated on the second day of hospitalization, and the mean appendix diameter of these 25 patients decreased significantly (p < 0.001) compared to the baseline (Table 2). The appendix was not visualized in 29 cases.

The main criterion of non-operative management of acute appendicitis was no signs of fecaliths in the appendix lumen; therefore, most cases were evaluated by a CT scan. If signs of fecalith were not clearly reported in the US exam, they were evaluated by a CT scan (Table 2).

Neither unresponsive cases nor complications (e.g. sepsis, ileus, perforation, and adverse drug events) were observed during the antibiotic treatment. Initial success rates were 100%. Readmission to the hospital was observed in five cases at the first, second, seventh, 14th, and 20th months of post-non-operative treatments, and they were subsequently treated laparoscopically. Histopathologic evaluations have revealed that no perforation signs were recorded in the specimen.

## Discussion

Pediatric appendicitis has a high perforation rate, and removal of the appendix is a conventional surgical operation. Therefore, appendectomy is the first choice of treatment in children. However, surgical interventions and general anesthesia have some inevitable complications (e.g. bleeding, ileus, surgical site infection, and pneumonia). For these reasons, in recent years, non-operative management has been preferred in some cases of acute appendicitis [17]. The basic hypothesis is that other acute appendicitis-like conditions (e.g. uncomplicated diverticulitis, salpingitis, and necrotizing enterocolitis) regress with antibiotics with a high success rate, especially when the medical treatment is started early [18]. Few studies have addressed non-operative management for acute appendicitis among pediatric patients, while this is a well-known option in the adult patient population [19].

Previous studies have demonstrated widely different success rates. These varied results might be due to patient selection criteria and antibiotic therapy protocols [2,4-16]. Antibiotic selection, antibiotic duration, and time for IV/per oral route have also been attracting research interest. A varied ratio of overall success is presented in the literature by the studies regarding children being managed non-operatively. The overall success rate in our study is higher than many studies in the literature. Among those studies, it is seen that the overall success rate was higher in studies where the patients were with short symptom duration (<36 hours) [4,14,15].

In this study, we reduced the symptom duration between the onset of complaints and admission (<24 hours), and we required additional criteria such as the patients to be “fever-free” at the initial examination. Being fever-free at the time of admission is an important sign of a non-complicated inflammatory period. This approach provided early antibiotic initiation and suppressed the inflammatory process. To date, meta-analyses are demonstrating that being fever-free at the time of admission is not an inclusion criterion for non-operative management [20,21]. Similarly, early antibiotic initiation has been reported to cause low recurrence rates of non-operative treatment [4,14,15].

The inclusion and exclusion criteria for non-operative management have been determined with/without fecalith and appendix diameter in imaging studies [4,7-9,14,15]. One of the main criteria in our study was no signs of fecaliths in the appendix. Unlike in previous studies, we performed a CT scan in 43 (79.6%) of the cases in our series. This is because, in the US examination, only 25 (46.2%) appendices were detected and verified without fecalith in the imaging studies. CT scan has high sensitivity and specificity rate for the diagnosis of acute appendicitis; however, the routine usage of CT scan is not recommended due to the high radiation exposure. The reduction of ionizing radiation has provoked the increased usage rate of CT year on year [22,23]. Sometimes CT scanning may be the first choice of radiologic evaluation for undiagnosed patients and obese children. The usage rates of CT imaging for the diagnosis of acute appendicitis vary according to clinical practice, surgeon preference, and institutions. The average rate is reported as 30-40% [24-26].

In some studies, to decide on non-operative management, the appendix diameter has been taken into consideration. It has been reported that the appendix diameter should be ≤9, ≤10, and ≤11 mm in various studies [7,9,15,27]. In the current study findings, we did not consider appendix diameter. In contrast, the appendix diameter was found higher than 10 mm in 17 (31%) patients, and they were treated non-operatively. However, the cut-off value of appendix diameter for non-operative management remains controversial. Also, we have determined that during the clinical improvement period, the appendix diameter decreases (p < 0.001). A critical evaluation was that acute uncomplicated appendicitis is suppressed with antibiotics. During the recovery period, among patients that responded, inflammatory signs (WBC and CRP) also decreased significantly relative to initial values. Based on this finding, we might update our approach when evaluating uncomplicated appendicitis in children.

The selection of antibiotics (e.g. cephalosporin, carbapenem, and β-lactam) and the duration of the prescription/therapy might differ among the clinical series [4-16]. Antibiotic duration for IV and oral administration has been reported to vary in the earlier reports. In our series, we preferred triple and narrow-spectrum antibiotics by IV route administered in the hospital for five days. The duration of antibiotic therapy was longer than the other reported series. Even in the early responding treatments of cases, IV treatment was completed in five days, as reported earlier.

A retrospective analysis reported that the antibiotic treatment was first applied in the emergency department and was provided to be used at home for two or three days in the total course [26]. The same analyses have reported that the success rate of their treatment was 58-99%. In our study, the positive responses of all cases to the treatment might be a result of the long-term usage of antibiotics.

The case numbers and follow-up periods of the literature studies were evaluated similarly. For long-term results, follow-up periods between six months and 4.3 years were reported. Besides, it has long been established that recurrences are the main factor in the success rate in the follow-up period. The early failure rate of these studies was between 1.2% and 41.6%, and the long-term failure rate was 8-42% in children [2,4-16,20]. There was no early failure case in our study; however, the long-term failure rate was 9% due to five recurrences of appendicitis. A meta-analysis of previous studies reported that the rate of appendectomy due to recurrence appendicitis was 18-42% within a one-year follow-up period [27-30]. Therefore, we included cases that have a follow-up period of at least two years. The mean follow-up period was 42 months in our study, whereas a small number of studies had a longer follow-up period than ours. Moreover, half of the published studies include less than 54 cases.

The main limitations of this study are that it is a single-center, retrospective, and uncontrolled study. Another limitation of our study is the longer duration of IV antibiotic therapy (five days) in the hospital. However, this can be interpreted as the learning curve of our clinic. In our current practice, we hospitalize patients for two or three days for IV antibiotic therapy.

## Conclusions

In conclusion, in this observational study, we found that non-operative management in children for acute uncomplicated appendicitis in selected cases is a safe and effective treatment method. Based on our findings, we propose that the success rate of non-operative management for clinically and radiologically proven acute appendicitis cases could be improved by applying two significant treatment criteria, i.e., less than 24 hours of symptom duration and fever-free at the time of admission.
